RETRACTED

# Mental Writing and Mental Health and Cultural Identity in Doris Lessing's Science Fiction

**DOI:** 10.1155/2022/2215829

**Published:** 2022-08-27

**Authors:** Yuhuan Liu

**Affiliations:** School of Foreign Languages, Changchun Institute of Technology, Changchun, China

## Abstract

As one of the most outstanding female writers in post-war Britain, Doris Lessing, winner of the Nobel Prize for Literature, has a strong spirit of the times in her works. In order to further understand the characteristics and spirit of the times in Doris Lessing's novels, Doris Lessing's science fiction is taken as the research object in this study, through in-depth research on novel storytelling, philosophical psychology, thematic forms, etc., from the perspective of emotional psychology model, to deeply analyze the characteristics of psychological writing, mental health, and cultural identity in their science fiction. Doris Lessing's science fiction reflects the political, cultural, and historical background of the times, and on this basis, it reflects humanitarian concerns through characters' psychological writing and cultural identity. It is shown in the results of the study.

## 1. Introduction

Doris Lessing (1919–2013) was one of the most outstanding female writers in post-war Britain. In 2007, she was awarded the Nobel Prize for Literature. Her works always have a strong background and characteristics of the times. In her writing, she uses the power of doubt, imagination, and enthusiasm to examine the era of divided civilizations in the twentieth century with different characters. Her works have a wide range of subjects and involve many types of content, especially the 20th-century turbulent social background and the description of reality, which vividly reflects the characteristics of “cultural identity exploration” [1]. The five-part novel *Canopu*s (1979–1983) is the representative work of Lessing's science fiction and an important part of its entire creation, depicting the space inhabitants in various terrible disasters and sufferings in the evolutionary segment of the universe (especially the fringe group) cultural identity and other living conditions. The work reflects the real content in the form of science fiction, reflects the plight of contemporary human existence and reflects Lessing's worry about the entire world civilization and the future destiny of mankind. It is a series of works that combine ideology and artistry. As a famous contemporary female writer, Lessing has been highly valued by critics, but the academic circles at home and abroad are relatively cold to Lessing's self-proclaimed space novels. In general, the research on space novels is mainly carried out from the aspects of overall commentary, philosophical psychology, thematic form, etc., few scholars discuss the cultural identity issues, and these works urgently need more attention [2].

RETRACTED

This article takes Doris Lessing's science fiction as the starting point and focuses on examining the psychological writing characteristics and cultural identity embodied in her novels through the introduction and analysis of the characteristics, mental health, and creative background of the novels. At the same time, on this basis, with the help of an emotional and mental model, even her science fiction reflects the political, cultural, and historical background of her times [3].

## 2. Literature Review

Lessing's science fiction has been widely concerned since its inception, and there are different voices in the literary world [4]. Literary critics such as Tylets, V. G. have argued that, “Despite some admirable qualities of Lessing's early writing career, I don't think her writing over the past fifteen years is readable. It's all fourth-rate science fiction.” [5]; As one of the few talented English-language writers of this century, why did Lessing continue to write science fiction that confuses and frustrates her loyal readers? He believed that people could not get lessons on Lessing's planet 8, but rather missed the realistic Lessing's concern for society and humanity. On the fourth day after the Nobel Prize Literature Committee announced the award of the Lessing Literature Prize, some scholars said that their first reaction after hearing the news was “This is a victory for science fiction!” *Canopus: The Archives* helped science fiction gain mainstream literary attention [6]. Lessing was an important science fiction writer from the 1970s to the 1980s. She argues that their *Canopus in the Southern Ship Galaxy: The Archives* series of novels demonstrates the importance of contemporary science fiction features [7].

AE León and others believe that almost all of Lessing's works have become the object of discussion by scholars. They analyzed Lessing and her works from different perspectives and with different theories. The research focuses on the works of the first and second stages such as *Golden Notes* and *The Weeds Singing*. Since the beginning of the 21st century, foreign countries have attached great importance to the comparative study of Lessing and her works and the works of other writers, and put her works into the context of the continuation and development of the literary history tradition and the feminist theoretical tradition to conduct holistic, comprehensive and dialectical research. In a word, foreign Lessing research started earlier, the research was relatively systematic and in-depth, and the research results were fruitful. A group of research experts appeared. Their research results strongly promoted Lessing research in the world and laid the foundation for domestic Lessing research [8].

RETRACTED

Science fiction plays an important role in Lessing's writing career, and she “enjoys writing science fiction, although the first few are difficult and painful.” Lessing's science fiction novels “are very different from her previous work in both form and content.” Her sci-fi work begins with *Briefing for a Descent into Hell* (1971), an “inner space novel” without a general storyline, mainly the protagonist's frantic hallucinations; it tells the story of a schizophrenic the patient who wanders the heavens and the Earth in fantasy, as if going through hell and witnessing all kinds of strange sights; it “opens up a new change in the form and narrative of Lessing's novels” [9]. Followed by *Memoirs of a Survivor*, Rodrigues, and others believe that the background is a future world that is about to collapse, and describes the pessimism and despair of a middle-aged woman who has experienced war and disaster as she witnesses a civilized society moving toward violence and destruction. Lessing “interweaves current facts with the future so serendipitously that we slip across boundaries into the future world without even noticing it.” These two mainly focus on the inner world of people. Rodrigues and others believe that the five-part novel *Canopus* focuses on the vast space universe, depicting a fragment of the evolution of the planets in the vast galactic empire. Several representative planets such as Sirius, Canopus, Pudiola, etc. are powerful, fighting with each other, with many contradictions, plundering and aggressing weak planets such as Shikasta, which is facing civilization regression, cultural decline, ecological deterioration, catastrophic issues like Doomsday. Lessing is pointing out the evils of the times and predicting future human disasters. There is basically no objection that these seven novels are science fiction [10].

## 3. Emotional Mental Model Based on Crowd Evacuation

### 3.1. Crowd Motion Modeling

#### 3.1.1. Roadmap Global Path Planning Method

In order to better simulate the crowd movement behavior in complex situations, this study uses the roadmap method to plan the complex environment as a whole in the preprocessing stage based on the crowd movement scene information, and generates a scene-based path network to find an optimal global situation for individual movement path. The process is mainly composed of two stages: the path construction stage and the path query stage [10].

RETRACTED

#### 3.1.2. RVO Local Obstacle Avoidance Algorithm

In the crowd path planning algorithm, the RVO algorithm is based on the geometric method and improves the traditional VO algorithm. By adjusting the movement speed of the individual, it can effectively avoid the collision between any individual A and B in the scene. The algorithm reduces the offset degree of speed, and ensures the avoidance of local obstacles without jitter between groups. The algorithm principle is shown in Figure 1.

### 3.2. The Emotional Infection Model

The influence of emotion on group movement behavior cannot be ignored. A large number of domestic and foreign scholars have conducted in-depth research on emotional infection, and according to the different internal infection mechanisms, they are mainly divided into two types: the emotional infection model based on thermal diffusion mechanism and the infection-based infection model. An emotional infection model of pathogenesis, as shown in Figure 2.

The ASCRIBE model is a typical thermophysical dissipation-based model proposed by VU University, which is based on individual interactions, and each individual has specific expressive power and sensitivity for the individual infection process. The model mainly defines five parameters, and all parameter values are between (0, 1).

The infectious disease model is based on the theory of physiology, mainly studies the transmission process and laws of disease outbreaks, and predicts its development trend. In recent years, this model has been widely used in the fields of social event turbulence, real network information, rumors, and emotional information dissemination between individuals. Based on the theory of infectious diseases, constructed an emotional infection model based on the mechanism of infectious diseases to study the emotional transmission and infection process between groups [11].

According to the infectious disease theory, the SI model divides the population into two main types (Figure 3): susceptible individuals (S) and infected individuals (I). During the spread of the disease, the infected individual will infect the surrounding susceptible population with a certain probability, and once the susceptible individual is infected with the virus, it will immediately become an infected individual and will never be cured [12].

In the SIS model (Figure 4), the population is similarly divided into susceptible individuals (S) and infected individuals (I). However, unlike the SI model, the SIS model further refines the transmission rules of the population. Infected individuals can become susceptible individuals through treatment, but there is still a certain probability of re-infection with the virus, and will not be permanently immune to the infectious disease [13].

RETRACTED

Different from the above infectious disease models, the SIR model divides the population into three types: susceptible individuals (S), infected individuals (I), and immune individuals (R). Among them, susceptible individuals have not yet been infected with the disease but have a certain probability of being infected with the virus [14], while the infected individual has already carried the virus and has a certain probability of infecting others, but at the same time has a certain probability of being cured and obtained permanent immunity, and eventually become immune individuals, while the immune individual develops antibodies to the infectious disease and can no longer be infected, as shown in Figure 5.

The SIRS model also divides the population into three types: susceptible individuals (S), infected individuals (I), and immune individuals (R), but unlike the SIR model, the immune individuals in the SIR model are permanently effective, while in the SIRS model, the immune individuals may become infected again by becoming infected with the virus [15], as shown in Figure 6.

### 3.3. Heterogeneous Emotional Infection Model for Crowd Evacuation Simulation

#### 3.3.1. Method Overview

The input of the method is the initialization of the scene model, emotional infection, and individual position information, and the output is the simulation effect of crowd movement. After initialization, our method mainly includes emotional infection and crowd movement [16].

#### 3.3.2. The Degree of Emotional Panic based on Characteristics

Emotion is a psychological reaction that accompanies people's feelings, cognition, and behavior. People can infect emotions by perceiving the emotional information of others and changes in the external environment, but differences between individuals will lead to different infection effects. Gender affects the intensity of an individual's emotional infection. Compared with men, women are more sensitive to emotions; and the differences in individual emotional infection are related to personality characteristics. Some individuals are more easily affected by surrounding emotions, while others are difficult to be affected [17]. The older the individual, the richer the life experience they have, which enables them to better regulate their emotional responses, pay more attention to positive emotions, and be less affected by negative stimuli. In the process of contagion of panic among the population, this study mainly considers the influence of three factors: personality, gender, and age. The factors within each factor are shown in Figure 7.

Personality is mental health that distinguishes people from others in terms of cognition, behavior, emotion, attitude, etc. Individuals with different personalities respond differently to emergencies. The OCEAN model proposed by the most commonly used personality model, which is described from five aspects: openness to experience, conscientiousness, extraversion, agreeableness, and emotional stability, also known as the FFM big five classification model. Its personality characteristics are shown in Table 1.

RETRACTED

From Table 2, in terms of gender, males and females have different emotional expressions and responses to the same external stimuli. In the process of emotional infection, women are more sensitive to the emotional impact of others, better at expressing and responding to emotions, and more likely to become emotional [18].

This chapter proposes a heterogeneous emotional contagion model based on Durupinar. In this model, adding the concept of group, the members of the group are more prone to emotional contagion, while the probability of emotional contagion between members of the group is small; using age the three characteristics of gender and personality specialize the individual to calculate the degree of emotional panic of the individual as shown in Table 3.

The number of infected people in different groups of heterogeneous and homogeneous models is also compared and analyzed, and the results are shown in Figures 8–10. Initially, in the heterogeneous model, only the individuals in the circle group were infected with emotion, and the rest of the groups were not infected; but in the homogeneous model, the individuals in all four groups were infected [19]. As the emotional infection time increased, it was only after 15 seconds that the rest of the individuals in the heterogeneous model in a different group from the round individuals began to infect emotions. The experimental results show that grouping has an impact on emotional contagion, and it is easier for members of the same group to influence each other to reduce the differences between each other, while members of different groups influence each other more slowly. However, when an individual in a group who wasn't emotionally infected became emotionally infected, the rate of infection in that group accelerated.

### 3.4. Spiritual Ecological Thought in Lessing's Science Fiction

#### 3.4.1. The Alienated Spiritual World

The human spiritual ecological crisis is different from the natural and social and ecological crisis. It is an internal and deep crisis. The progress of science and technology and the abundance of materials have not only brought prosperity and enjoyment to human beings, but also led to the continuous deterioration of the living environment and the degradation of human organisms, which are reflected in the spiritual space of human beings: the desire to pursue, the material satisfaction brings the anxiety of the mind [20], the shrinking of the soul and the disappearance of the once beautiful and sincere emotions. Joyce once said: “Modern man has conquered space, conquered the Earth, conquered disease, conquered ignorance, but all these great victories have only turned into a tear in the melting pot of spirit!”③In *Shkasta*, it refers to the “Shkasta” of the Earth, which became the colony of the three major empires of the Milky Way, “Shamat,” “Sirius” and “Canopus,” Canopus spreads kindness in Shikasta, the idea of harmony, where Shamat plunders wildly, and Sirius conducts species experiments here. Under the rule of the three major planets, Shikasta, who lost the flow of telepathic material, developed “mental degeneration,” and they became irritable, fierce, vain, and greedy. Shikasta declined to a social state of backward spiritual civilization and turned into a spiritual wasteland, which almost led to the destruction of the entire planet. Only the development is correct, but some problems caused by development are often ignored [21]. Disasters are brought about by rising seawater, melting of icebergs in the Arctic Ocean, snow disasters, and environmental pollution. ① The main culprit leading to these natural disasters is the degeneration of human thought, which is fully reflected in the article *Shkasta*. Nature is a mirror of human beings. When the natural ecology is destroyed, the spiritual ecology of human beings will also be out of balance. The relationship between man and nature determines the essential connotation of the relationship between man and man, man and self. In Lessing's science fiction works, we see the increasingly alienated human spiritual world. Here, life is shrinking, humanity is gradually lost, ethical and moral consciousness is fragile, and human beings are almost reduced to a state of walking dead.

RETRACTED

#### 3.4.2. Return to Nature, Return to Self

From the characters in Lessing's science fiction, we can see her ecological concept of advocating equality of all things and protecting nature. After his marriage to Ellie Eas, Ben Aita's thoughts have changed a lot. He dismantled three-quarters of the army and sent them home to dig ditches and cultivate the land to improve their living standards; allow women they visited zone three; let the children go to zone three to learn advanced ideas and concepts. Ben Aita's change in attitude towards people and things was under the subtle influence of Ellie Iss, and it was a conscious adjustment behavior, because all lives in the kingdom should be honored: the thinking man experiences the will to all life as he must fear his own, and he experiences other beings in his own life. ① Ellie Eise also saw her own shortcomings in Ben Aita, she was too rational and lacked an impulse. She returned to zone three, only to encounter indifferent banishment, her sister became queen, and she was imprisoned in the suburbs. It was during these days that Alice Ease, who was forced to give up her status as a queen, her wife's obligations, and her mother's responsibilities, lived the simplest life in nature. I gained strength and courage from nature and went to zone two, which I have always dreamed of. In this interracial marriage, Ellie Eith found her own shortcomings, found herself in nature, and gained a new life. Ness proposes that the maturity of the self needs to go through three stages: from the individual to the social self, and then to the ecological self [22]. The process of self-realization is the process of interaction between human beings and nature. People constantly expand the scope of objects of self-identification, narrow the differences with other existences, and integrate with nature to achieve the highest state of harmonious coexistence.

Everyone should see themselves as an organic part of the ecological whole so that a sense of identification with others and with natural beings expands: “It is only when people live in a soil, water, plant and protectionism is only possible in a community in which animals are all members and assume a civic role; in a community in which each member is interdependent, each member is entitled to a place under the sun.” “② Nothing in nature exists in isolation, and we should treat all life with an attitude of equality, respect, and cherishment because harming anything in nature is harming ourselves. In *Crack*, the men are punished for wreaking havoc on nature—their homes are destroyed in the wind. This sudden disaster made them temporarily stop fighting each other and face the crisis of survival together. The two sexes began to have substantial contact. They knew and understood themselves through each other, and they began to slowly integrate in their lives. They recognized each other's differences and understood that the two sexes should tolerate and help each other [23].

## 4. The Cultural Identity of the Diaspora in Lessing's Space Fiction

### 4.1. The Confusion of Mixed Identities of the Diaspora

#### 4.1.1. Ellie's Mixed Identities and Confusion in *Marriage*

Ellie in *Marriage* is a typical representative of the diaspora in Lessing's space novel *Canopus* series. After she was ordered to marry King Ben of zone four, she began a journey of diaspora, gradually moving from the center of society to the fringes; and the order of marriage in zones four and five terminated her diaspora life in zone four and was forced to go into exile again. The dual existence of diaspora “creates the duality and hybridity of the cultural identity of the diaspora.” ① The diaspora Ellie lives in two cultures, with mixed identities, making it difficult to unify. The mixed identities make Ellie's identities contradictory, and she is confused and disturbed by it. Clearly, in Ellie, mixed identities are evident. In the migrations and diasporas, Ellie travels in different regions, ethnic groups, races, cultures, and languages, which is accompanied by the fission of her identity, the contradiction of mixed identity, the alienation of culture, the pain of self-tear, identity recognition confusion and uncertainty about where they belong. Obviously, Ellie's identity changes with time and space, and is affected by the situation she is in, indicating that “the self is the product of some special interactions, and the individual's abilities, attitudes, and behaviors will change with the changes of the surrounding people.” ② Who is Ellie whose identity is changing? She is everything and nothing. Ellie's hybrid cultural identity is unmistakable. None of these cultural identities are pure. One identity has an influence and effect on the other, and conflicts arise all the time.

RETRACTED

#### 4.1.2. The Mixed Identities and Distresses of Other Imperial Diasporas

Mixed identities haunt Ellie, as well as the scattered imperial emissaries and spies in Lessing's space novel *Canopus*. There are many messengers sent by the space empire Canopus to the colonized planets, such as Johe, Korossi, and Nassar; members of the leader group such as Amy Bean I and II of the space empire Sirius also often visit the colonized planets; Deora also often sends representatives such as Krogul to colonize planets; this does not include spies lurking in various countries. The envoys or spies of the empire lived in foreign places for a long time or frequently traveled to and from their homes and foreign places, whether it was voluntary or forced, “dispersion” became their living state.

The mixed identity and uncertainty of identity of the diaspora of the space empire are also displayed in Mary in *The Weeds Sing*, Martha in the *Violent Children* five-part novel, and the author himself. This mixed cultural identity makes it impossible for the imperial diaspora to distinguish between “this” and “that,” and often struggle with the confusion of “this and that” and “neither this nor that.” Sandwiched between imperial culture and colonial culture, the imperial diasporas such as Queen Ellie of zone three, Sirius Senior Leader Amy Bien II, Canopus messenger Johe, Korossi, Nassar and other imperial diasporas seem to all agree with these cultural identities, and can not agree, can not be sure, and anxious. With mixed cultural identities, they experience the collision of heterogeneous cultures and the resulting division and pain of cultural identities, but they cannot fully integrate into any of them to achieve cultural harmony. These diasporas are very at a loss, living in the predicament of living on the edge, mentally anxious, and suffering. Since they are not sure “who I really am,” in them, we can see their sense of rootless wandering, entangled fear and confusion, pain and confusion in the cultural conflict. This state of living in cultural conflicts and gaps has led to the division of subjectivity, the anxiety of identity, and the confusion of positioning of these imperial diasporas, and their self-identity cannot be confirmed in a continuous cultural situation [24].

RETRACTED

### 4.2. The Loneliness of Cultural Alienation of the Diaspora

#### 4.2.1. Alienation and Cultural Alienation

Both Asian-African diasporas and imperial diasporas are in the middle of heterogeneous cultures, alienated from the culture of the mother country, and difficult to integrate into the culture of the place where they migrated, resulting in a sense of alienation. At the same time, they experienced the mental pain caused by cultural alienation. On the one hand, they were sad because they could not get close to their hometown, and on the other hand, they were distressed because they could not integrate into life in the place where they lived. The diaspora gradually finds that they are separated from their home country and unable to integrate into the place where they live. They are forever in a state of wandering, resulting in a “feeling of ‘rootless'” and “spiritual exile.” ④ Cultural alienation has caused the diaspora to lose their orientation and sense of belonging, and finally, make them fall into an identity crisis. Therefore, the diaspora usually have a kind of confusion: “Who am I?” “Where am I going?” With their broken national memories, they wander on the edge of multiple cultures, and in the new cultural situation, their identities are constantly split, and they are always in the identity. Suspended state, felt deeply anxious and bewildered by this.

#### 4.2.2. Bicultural Alienation of Diaspora in Lessing's Space Novels

The conflict between Ellie and Ben in *Marriage* shows her alienation from the culture of zone four. After marriage, Ellie and Ben continued to work together, and the two cultures gradually merged. However, due to differences in life experience, way of thinking, and behavior, there were constant conflicts between them. In the work, the marriage of Ellie and Ben is to produce offspring to integrate the cultures of the two zones, but the different attitudes and ways of the two toward sex interpret the conflict between the two. Ellie from zone three and her nationals understand the basic skills of sex and pay attention to the emotional communication and feelings during sex. But Ben and his people of zone four are vulgar, “have a repulsive overheated sensuality” and in their sexuality, care only about possession and not about women's feelings. Ben is accustomed to violently possessing women, and he often brutally assaults women captured in battle, finding satisfaction in their fright, crying, cursing, and struggles. When Ben finished his first sex with Ellie in the same domineering and rude manner, there was absolutely no love between the two that Ellie expected. Ellie neither rejected nor cried Muran also surprised Ben, and he did not gain the slightest sense of conquest, feeling like a rude man. Ben's demeanor showed that he was a rude, brutish savage with no taste for fun, while the men in zone three were warm, caring, empathetic, civilized people in Ellie's recollections. Ben's sexual attitude and behavior are obviously different from those of men in zone three. In Ben's “terrible country,” Ellie can only allow Ben to “violate” in any way, but Ellie “cannot stop” him. But it was really difficult for her to accept it, so she could only bear it silently. Although Ellie and Ben's emotional lives are constantly harmonious, the two different sexual concepts and behaviors reflect their contradictions and the conflict between the two cultures. Cultural conflict will inevitably “cause a crisis of cultural identity.” Ellie rejects this crude and backward culture of zone four from the bottom of her heart, and Ben's “strong hatred for Ellie finally culminates in raising his hand to beat her.”

RETRACTED

### 4.3. The Rootless Confusion of Exiles

#### 4.3.1. The Home of the Diaspora

Writer Naipaul is a rootless diaspora in constant search for himself in order to confirm his identity. However, he was alienated from the Indian culture of his home country and could not integrate into Trinidad, his birthplace. He rushed to the imaginary homeland of England but could only linger on the edge, and returned to India to find his roots but left disappointed. He gradually lost himself in the change of time and space in his search for his homeland, and increasingly became a “rootless person” who had a nationality but no motherland, a bloodline but no affiliation, and achievements but no clan applause.” Naipaul was always on the road in order to reconstruct himself, never reaching home. With nowhere to go, he is always anxious, confused, and uneasy. He does not know where to go, where to go, and he cannot even confirm who he is and who he will be. Lessing, who was once scattered in Asia and Africa, and later settled in London, had a similar experience with Naipaul in the search for himself and his home, and the anxiety and confusion of self-lost. Lessing was born in Iran, grew up in Southern Rhodesia, Africa, experienced two short-lived marriages, returned to London, and returned to Africa several times. She and the characters in her novels are always on the road looking for a home to live in, but they do not know where to be home and where to go. This state of not arriving at home and not confirming herself makes her and the characters in her works always in mental anxiety and confusion. The search for the road and the loss of self are also prominently reflected in Lessing's African-background novels and science fiction such as *Canopus*.

#### 4.3.2. The Wandering of the Homeless

The imperial diaspora in Lessing's space novel series lived in a foreign land and longed for their homeland. Due to their long-term exile, they had no fixed place to live, and finally lost their homeland and wandered around. It is their grief, a sign of their lost identity, and an important theme in the representation of postcolonial fiction. Diaspora means “a new geographic location of identity”; Saffron, Cohen, and many other sociologists believe that “connection with one's homeland is critical in identifying diaspora and diaspora subjects.” Diaspora is closely related to places such as region and homeland. For the diaspora, who often span two or more locations, home “is both an actual geographic location and an imaginary space.” The diasporas such as Ellie in Lessing's space novels are basically what Mei Xiaoyun called “rootless-rootless.” They are alienated from the culture of their home country and cannot identify with the culture of the guest place. They are true wanderers without roots. For them, the homeland of the motherland has drifted away, and although they have a temporary shelter in the place of emigration, it is not their home. They lost their homeland not only geographically but also spiritually and culturally, and became exiles with nowhere to go.

## 5. Conclusion

Doris Lessing, Britain's most outstanding female writer after World War II, has experienced almost the entire 20th century, witnessing the changes and turmoil of the times. Having lived in Africa once, she has witnessed the injustice of colonial society and the difficult life of the colonized, experienced the life of the marginalized diaspora, suffered the confusion and crisis of identity, and has been pursuing the identity and construction of cultural identity. Lessing has her own sensory experience of life, profound insights into social issues, and a unique perception of life. The experience of exile and the experience of others made her pay special attention to the living conditions of human beings (especially the marginalized groups in society) and the future of human beings. The maverick Lessing is a stubborn adherent of authentic survival, and writing is the artistic expression of this way of life. The wandering life situation and sensitive female experience have made Lessing's unique creative concept and writing style. Lessing not only inherits the tradition of British realism novels, but also constantly innovates boldly, breaking through themes and genres, transcending the conflicts and divisions of reality, and embodying the distinctively modern and postmodernist characteristics of mental health and the characteristics of the times and unique styles. Lessing's creative subjects are diverse, involving politics, colonization, race, women, religion, war, ecology, technology, identity, and many other themes of the entire era. Lessing has the spirit of the times. Through her works, she can gain insight into the social reality of a century. This is an important reason why Lessing's research is highly valued. Undoubtedly, Lessing's research has important implications for understanding twentieth-century society, the west, and British literature, culture, history, and politics.

RETRACTED

## Figures and Tables

**Figure 1:** Principle of RVO algorithm.

**Figure 2:** Emotional psychology.

**Figure 3:** Principle of SI model propagation.

**Figure 4:** SIS model propagation principle.

**Figure 5:** Principle of SIR model propagation.

**Figure 6:** Principle of SIRS model propagation.

**Figure 7:** Factors affecting the degree of emotional panic.

**Figure 8:** Group 1: Round individuals.

**Figure 9:** Group 2: Rhombus individuals.

**Figure 10:** Group 3: Square individuals.

**Table 1:** The main content of the model.

Specific character	Main features
0	Imagination, creative power
*C*	Responsible and persistent
*E*	Good communication, active
*A*	Warm-hearted and helpful
*N*	Anxiety, impulse

**Table 2:** Personality panic factor division.

The value of *per*	Personality classification	Main features	The value of *μ*_*p*_	The value of *σ*_*p*_
[0, *per*_1_]	Sensitivity pattern	Impulse, uneasy	0	0.2
(*per*_1_, *per*_2_]	Stable type	Easy-going, calm	0.45	0.3
(*per*_2_, 1.0]	Calm type	Calm, conservative	0.15	0.2

RETRACTED

**Table 3:** Emotional value and emotional state division.

Emotional state	The value of *e*
No panic	0
Mild panic	(0, 0.3]
Moderate panic	(0.3, 0.8]
Severe anxiety	(0.6, 1.1]

## Data Availability

The labeled data set used to support the findings of this study is available from the author upon request.
